# Evaluation of post-COVID mortality risk in cases classified as severe acute respiratory syndrome in Brazil: a longitudinal study for medium and long term

**DOI:** 10.3389/fmed.2024.1495428

**Published:** 2024-12-18

**Authors:** Nádia Cristina Pinheiro Rodrigues, Mônica Kramer de Noronha Andrade

**Affiliations:** ^1^Departamento de Epidemiologia e Métodos Quantitativos em Saúde/Escola Nacional de Saúde Pública Sérgio Arouca/Fundação Oswaldo Cruz, Rio de Janeiro/Brasil and Departamento de Epidemiologia/Instituto de Medicina Social Hesio Cordeiro/Universidade do Estado do Rio de Janeiro, Rio de Janeiro, Brazil; ^2^Programa Academico de Tuberculose/Faculdade de Medicina/Instituto de Doenças do Torax/Hospital Universitário Clementino Fraga Filho/ Universidade Federal do Rio de Janeiro, Rio de Janeiro, Brazil

**Keywords:** COVID-19, COVID-19 vaccines, severe acute respiratory syndrome-related coronavirus, mortality, survival analysis, longitudinal studies

## Abstract

**Background:**

There are few studies in the literature evaluating post-COVID mortality in Brazil, along medium and long term, especially in those who presented severe clinical disease.

**Objective:**

This study aims to investigate the factors associated with post-COVID mortality of severe acute respiratory syndrome (SARS) cases from 2020 to 2023 in Brazil, along medium and long term.

**Methods:**

Retrospective cohort study using notification data of SARS classified as COVID-19 from the Brazilian National Information System, “Sistema de Vigilância Epidemiológica (SIVEP),” during the period 2020 to 2023. Data included demographics, comorbidities, vaccination status, number of COVID-19 vaccine doses, city of residence, and survival outcomes. Classic Cox, Cox mixed effects, and Cox fragility models were used to assess medium and long-term risks of dying post-COVID.

**Results:**

In the medium and long-term periods studied, 5,157 deaths were recorded out of 15,147 reported SARS/COVID-19 cases. Of these deaths, 91.5% (*N* = 4,720) occurred within the first year, while 8,5% (N = 437) after the first year. People without formal education, the older adult, had higher percentages of deaths in both periods. In the medium-term post-COVID period, the risk of death was reduced by 8% for those who had been vaccinated while in the long-term post-COVID period, the risk of death almost doubled for those who had been vaccinated. While in the medium term, there was a reduction in mortality risk for those who took two or three doses, in the long term the risk of death was greater for those who took one or two doses.

**Conclusion:**

The protective effect of COVID-19 immunization was observed up to one year after the first symptoms. After one year, the effect was reversed, showing an increased risk of death for those vaccinated. These results highlight the need for further research to elucidate the factors that contribute to these findings.

## Background

The COVID-19 pandemic has had a catastrophic impact on global health, with several factors influencing the risk of death among reported cases. Recently, in a Brazilian longitudinal study of mortality risk after COVID-19, the authors showed that the risk of death increased in different demographic groups and people with co-morbidities. Men, older people, blacks, those with a lower level of education, and those living in urban areas, especially from the state of Rio de Janeiro, faced a higher risk of death. Nevertheless, vaccination reduced death risk by around 20 and 13% in 2021 and 2022, respectively (1). All these findings were similar to other studies (2, 3).

The vaccines were therefore relevant tools for changing the COVID-19 scenario in the world. New technologies, including the m-RNA mechanism, have been used to develop COVID-19 vaccines. Studies on the efficacy and effectiveness of vaccines have been conducted to determine public health policy strategies for effective control of COVID-19 over time up to 2022 (4). According to the Centers for Disease Control and Prevention (CDC) Vaccine Adverse Event Reporting System (VAERS) (2023), out of 550 million doses of the SARS-CoV-2 vaccine administered, only about 0.0042% of serious adverse events were reported (5, 6). Long-term monitoring by VAERS has shown a lower frequency of reports of serious side effects related to mRNA vaccines (7).

However, few estimates of updated 2023–2024 vaccine effectiveness (VE) are available, but receipt of the updated COVID-19 vaccine provided approximately 54% increased protection against symptomatic SARS-CoV-2 infection compared with no receipt of the updated vaccine. Recently, CDC’s Advisory Council on Immunization Practices recommended updated 2023–2024 COVID-19 vaccination (monovalent XBB.1.5) for all persons aged ≥6 months to prevent COVID-19, including severe disease and CDC will continue monitoring COVID-19 VE, including against severe disease and for expected waning (8).

The Brazilian Immunization Program was quite strong until 2020. However, during the COVID-19 pandemic, there was a lack of organization of this program due to political problems and, consequently, weak national planning for the acquisition of vaccines and delay in distribution to the population. The new Plan only encompasses around 40% of the country’s population, failing to obtain the number of doses ideally needed to achieve immunity (9). As a result, the COVID-19 vaccination campaign was launched on January 17, 2021, and initially targeted high-risk groups only: health care workers, the older adult, and patients with comorbidities and vulnerable populations such as Indigenous, homeless, quilombos and border river population, prisoners. Three vaccines were authorization by ANVISA, one of them with emergence use authorization (SINOVAC/Butantan) and others, with definitive registration (AstraZeneca/Fiocruz e Pfizer). However, only Sinovac/Butantan (inactive virus) and AstraZeneca/FIOCRUZ (recombinant) were available when the beginning of the vaccine campaign. Later, the m-RNA vaccine group also became available (10).

Studies of post-COVID-19 mortality in a country with the demographic and social characteristics of Brazil offer a unique and valuable perspective that complements global evidence, providing crucial information for public policies and health strategies. Brazil is a huge country divided into five macro-regions: North, Northeast, Midwest, Southeast and South. In this scenario, there is great diversity in terms of economic, social, geographical, and cultural aspects, with significant inequalities between them. Factors such as level of education, access to health care, prevalence of comorbidities (such as diabetes, hypertension, and heart disease), and different lifestyles of remote and more vulnerable populations can influence overall post-COVID-19 mortality. Studying post-COVID-19 mortality in Brazil allows us to identify specific patterns that may not be observed in other contexts, helping to tailor public health interventions to vulnerable populations, such as the older adult, people with low education, and people with comorbidities.

Therefore, longitudinal studies will be important to identify the factors associated with medium and long-term mortality post-COVID-19 and should be conducted to improve public health policy.

This study aims to investigate the factors associated with the risk of post-COVID mortality of SARS cases from 2020 to 2023 in Brazil, along medium and long term.

## Methods

This is a retrospective cohort study using the notification data of Severe Acute Respiratory Syndrome (SARS) classified as COVID-19 by the Brazilian National Information System, “Sistema de Vigilância Epidemiológica (SIVEP)” from 2020 to 2023 (11) SIVEP data are publicly available and include all reported cases of SARS in the country (https://opendatasus.saude.gov.br/dataset). Brazil is a huge country with five regions, 26 states, 5,570 municipalities, and a population of 203 million.

SIVEP is used to track outbreaks of respiratory diseases, including influenza and COVID-19. SIVEP-Gripe coverage is nationwide and includes data from all Brazilian states. However, data coverage and quality may vary, with differences observed between states and municipalities. Information is collected from hospitals and health units that report cases of SARS, regardless of laboratory confirmation of the causative agent (12).

SARS is a condition in which a respiratory infection causes severe breathing difficulties and alveolar damage. It includes cases of influenza-like syndrome that progress with impaired respiratory function (13). The definition used by the Ministry of Health published in an official document to support health professionals, including for notification in the SIVEP, advises that hospitalized SARS cases or deaths from SARS should be considered regardless of whether the patient was hospitalized. It defines a case of SARS as: “Individual with Flu-like Syndrome who presents: dyspnea/respiratory distress or persistent pressure or pain in the chest or oxygen saturation less than 95% in room air or bluish color (cyanosis) of the lips or face” (14). Since all cases included in this study were collected from SIVEP and included only cases of SARS, the cases included in the present study refer only to patients with more severe respiratory pathology and therefore more fragile patients.

In the study’s early phase, a survival curve was constructed for individuals with SARS diagnosed with COVID-19 from 2020 to 2023 (Figure 1). To capture only deaths that are not directly attributable to COVID-19 from post-immediate hospitalization and discharge, our approach involved analyzing data exclusively from patients diagnosed with the disease more than three months from the symptoms. A previous study published by us investigated the role of COVID-19 immunization and other factors on mortality in the first three months after the first symptoms of COVID-19 (1). To determine post-COVID deaths included in this study, we collected information on the date of COVID-19 first symptoms and date of death (regardless of the cause of death). Only individuals with at least a three-month interval between the COVID-19 first symptoms and death were included in the study. The clinical case definitions from the National Institute for Health and Care Excellence (NICE) guideline (2021) (15) were not included in this analysis, because in this study we worked only with very severe patients with SARS, collected from SIVEP from 2020 to 2023.

**Figure 1:** Post-COVID-19 survival in Brazil according to COVID-19 immunization: at least one dose and number of doses, 2020–2023. Kaplan Meier survival analysis.

Visual inspection of the survival curve revealed a notable difference between vaccinated and unvaccinated individuals especially starting one year after diagnosis. As a result, two distinct periods were defined as the medium and the long term: the first covering three months to one year after diagnosis and the second extending beyond one year (Figure 1).

Survival and risk of death overtime were calculated considering the two post-COVID periods: the medium-term period encompassed the interval between three months and one year after the first symptoms of COVID-19; the long-term period encompassed all individuals whose death occurred after one year of the first symptoms of COVID-19.

It is important to emphasize that this research included all recorded deaths from SARS or other causes that occurred at least three months after the onset of symptoms, regardless of the length of hospitalization.

We gathered data on various parameters, including death status, state of residence, municipality of residence, date of first symptoms, date of hospitalization, date of death, age, older adult population (≥65 years), sex, race (white, black, yellow, mixed race, and unknown), years of study (zero, 5, 9, 12, >12, and unknown), type of residence area (urban, peri-urban and rural), hospitalization, COVID-19 vaccination status (at least one dose), number of doses of COVID-19 (ranging from zero to three) vaccine, the presence of any risk factor for COVID-19 (defined in SIVEP as individuals with any of the following conditions: postpartum woman, heart disease, diabetes mellitus, asthma, hematological disease, Down Syndrome, neurological disease, immunosuppression, liver disease, kidney disease, and obesity), in addition to each of these conditions collected individually. Data from the unknown category of variables were collected and described.

Relative and absolute frequencies were calculated for the predictors according to death status, as well as the means and standard deviations of age. Statistical tests (Chi-square and Fisher tests) were performed to compare the groups. Survival tables and Kaplan Meier curves were constructed to compare the survival experience in the different states, years, educational levels, races, genders, and age groups. *p*-values lower than 0.05 were considered statistically significant.

Kaplan Meier curve was built to describe the survival experience in vaccinated and unvaccinated groups, as well as according to the number of vaccine doses regardless of vaccine type.

The percentage excess of death was calculated for those immunized against COVID-19, comparing them with those who were not immunized. The following expression was used for the calculation (16):


$$\mathrm{Excess}\_\mathrm{percent}=\frac{\left(\mathrm{observerd}\_\mathrm{deaths}-\mathrm{expected}\_\mathrm{deaths}\right)}{\mathrm{expected}\_\mathrm{deaths}}*100.$$

Where Excess_percent is the percentage excess of deaths among immunized individuals; expected_deaths is the expected number of deaths among immunized individuals, considering that this is independent of the effect of COVID-19 immunization, and observed_deaths is the number of deaths observed among immunized individuals.

Classic Cox, Cox mixed-effects, and Cox fragility models were fitted to analyze the risk of death over time. The unknown category of the variables was only included in the models when there were at least 50 deaths in this category. The Classic Cox Model assumes proportional hazards with no unobserved heterogeneity. The Cox Mixed-Effects Model extends the Classic Cox Model to account for unobserved heterogeneity by including random effects (frailty terms), often used to model clustering in the data. The Cox Frailty Model is similar but specifically focuses on the inclusion of frailties (random effects) to capture unobserved individual differences in the baseline hazard, and it can be used to model heterogeneity in survival times across individuals (17).

In the Cox Frailty Model, the frailty effect is treated as a component of the hazard rate, with the idea that the failure risk of each unit within the group (county) is affected by a shared frailty factor. This model does not explicitly specify a distribution for the frailty effect, although the survival package assumes a Gamma distribution by default. In the Cox Mixed-Effects Model, there is an explicit specification of a random effect for the municipalities, which allows for greater flexibility. The estimate of the random effect is directly related to the variance of the random effect for the county, which reflects the variation between counties that cannot be explained by the observed covariates. In addition, the Cox Mixed-Effects takes a more formal approach to modeling the hierarchical structure of the data, allowing for more control over the structure of the model (17).

The specification of the models is detailed below.

The classic Cox-adjusted model included the following predictors: number of vaccine doses administered, age, sex, race, years of education, region, hospitalization, and risk factors.

The adjusted Cox mixed effects and Cox fragility models included fixed effects of the number of vaccine doses administered, age, sex, non-white (race), years of study, hospitalization, and risk factors, and the random effect of the municipality of residence.

To calculate the adjusted effects of COVID-19 immunization (people who have taken at least one dose of the vaccine), the same models were adjusted by replacing the variable “number of doses of COVID-19 vaccine” with the variable “COVID-19 immunization.”

The race variable was included in the models as a variable with three categories (white, non-white - categories black and mixed race, and unknown – categories unknown and yellow).

The interaction of race and schooling was tested. By including both race and schooling in the model, there is the possibility that these variables are correlated, especially in contexts where certain racial groups have more or less access to formal education. By testing this interaction, we would avoid the risk of multicollinearity in the model.

The Variance Inflation Factor (VIF) values were estimated in the classical Cox model to investigate the presence of collinearity between the independent variables. Model goodness-of-fit measures were calculated for all models.

The Intraclass correlation coefficient (ICC), Akaike Information Criterion (AIC), and the Bayesian Information Criterion (BIC) were estimated. ICC is useful to estimate the proportion of variance explained by the grouping structure (in this case, municipalities). AIC is useful when the goal is to find a model that minimizes information loss and is particularly suitable for prediction. BIC is an approximation of the Bayes criterion for the marginal probability of a model given the observed data, penalizing models with many parameters, being especially suitable when dealing with large volumes of data.

Martingale residuals for the classic Cox models and the Cox frailty models were calculated to investigate whether trends might exist.

The R-project software version 4.3.2 was used in the analyses.

This research project does not meet the requirements for projects that require ethical assessment as established by Resolutions 466/12 and 510/16 and therefore does not need to be submitted to ethical assessment by the Brazilian CEP-CONEP system.

## Results

Out of 15,147 SARS/COVID-19 cases, 5,157 deaths were recorded over the post-COVID period studied. Of these deaths, 91.5% (*N* = 4,720) occurred in the medium term while 8.5% (*N* = 437) in the long term.

The mean age was great for those who died (medium-term period: 64.82 vs. 55.16 for dead and alive, respectively; long-term period: 70.53 vs. 53.42 for dead and alive, respectively) (data no showed). In both periods, the percentage of deaths is higher for those who have been vaccinated against COVID-19 and for those who took one or two doses of the vaccine. People without formal education and the older adult showed higher percentages of deaths. The North and Northeast regions showed the highest percentage of death in the medium and long term, respectively. Those with any risk factors for COVID-19 had a higher percentage of deaths in both periods. Specifically, for diabetes, heart disease, and kidney disease, the mortality was higher in both periods, for neurologic disease and Down Syndrome it was higher in the medium term, and for liver disease, it was higher only in the long term period (Table 1).

**Table 1:** Distribution of predictors according to death status of post-COVID cases, Brazil, 2020–2023.

Predictors	Medium-term period		Long-term period	
	Deaths (%)	*P*-value	Deaths (%)	*P*-value
**Older adult**		0.0001		0.0001
Yes	2,652 (46.70)		304 (47.90)	
No	2068 (26.00)		133 (15.00)	
**Sex**				0.53
Female	1993 (34.10)		208 (29.50)	
Male	2,727 (35.10)		229 (28.00)	
**Race**		0.002		0.01
White	1997 (36.98)		209 (32.20)	
Black	221 (35.88)		16 (21.62)	
Yellow	50 (42.37)		0 (0.00)	
Mixed race	1,605 (33.65)		141 (28.09)	
Unknown	847 (31.15)		71 (24.82)	
**Years of study**		0.0001		0.0001
Zero	157 (50.65)		21 (55.26)	
1–5	498 (45.19)		60 (39.47)	
6–9	316 (38.40)		29 (29.90)	
10–12	482 (34.55)		36 (21.05)	
>12	272 (33.17)		21 (24.14)	
Unknown	2,995 (32.65)		270 (27.61)	
**Region**		0.0001		0.0007
North	374 (41.90)		30 (35.70)	
Northeast	968 (35.80)		94 (37.80)	
Southeast	2,220 (33.10)		242 (26.90)	
South	729 (37.40)		41 (29.50)	
Midwest	428 (31.40)		30 (19.70)	
**Area**		0.32		0.009
Urban	3,937 (34.61)		356 (27.70)	
Rural	172 (35.54)		13 (21.31)	
Peri-urban	10 (23.81)		1 (50.00)	
Unknown	601 (34.86)		67 (38.29)	
**Year**		0.0001		0.02
2020	2,150 (35.40)		202 (25.80)	
2021	2062 (33.60)		234 (31.70)	
2022	442 (36.10)		1 (50.00)	
2023	66 (35.30)		0 (0.00)	
**COVID-19 immunization**		0.0001		0.03
Yes	1,064 (38.60)		134 (33.60)	
No	2,989 (34.20)		277 (27.50)	
**Number of doses of vaccine**		0.0001		0.0001
Zero	3,704 (33.60)		309 (27.00)	
1	263 (37.30)		26 (42.60)	
2	542 (40.90)		85 (38.50)	
3	211 (36.40)		17 (17.90)	
**Hospitalization**		0.32		0.006
Yes	4,511 (34.63)		394 (27.84)	
No	85 (37.95)		25 (45.55)	
Unknown	124 (33.24)		18 (33.96)	
**Any risk factor**		0.0001		0.0001
Yes	3,694 (39.90)		310 (34.60)	
No	1,026 (23.50)		127 (20.20)	
**Heart disease**		0.0001		0.0001
Yes	2019 (42.06)		167 (37.28)	
No	913 (35.86)		56 (22.95)	
Unknown	1778 (28.45)		214 (25.75)	
**Diabetes**		0.0001		0.0001
Yes	1,532 (43.13)		129 (38.62)	
No	1,223 (36.65)		75 (24.27)	
Unknown	1965 (29.18)		233 (26.48)	
**Kidney disease**		0.0001		0.003
Yes	434 (54.80)		22 (50.00)	
No	1835 (37.27)		128 (26.78)	
Unknown	2,451 (30.99)		287 (28.67)	
**Liver disease**		0.09		0.04
Yes	57 (46.34)		7 (58.33)	
No	2063 (38.68)		139 (27.63)	
Unknown	2,600 (31.83)		291 (28.87)	
**Hematologic disease**		0.15		0.51
Yes	61 (45.19)		4 (36.36)	
No	2082 (38.89)		141 (28.03)	
Unknown	2,577 (31.68)		292 (28.94)	
**Immunodepression**		0.10		0.14
Yes	221 (42.34)		12 (40.00)	
No	1956 (38.59)		134 (27.18)	
Unknown	2,543 (31.66)		291 (29.10)	
**Neurol disease**		0.0001		0.06
Yes	363 (49.25)		22 (40.00)	
No	1888 (38.02)		133 (27.71)	
Unknown	2,469 (31.17)		282 (28.54)	
**Down syndrome**		0.01		0.19
Yes	34 (54.84)		2 (66.67)	
No	2097 (38.71)		142 (27.79)	
Unknown	2,589 (31.79)		293 (29.04)	
**Asthma**		0.57		0.45
Yes	129 (37.39)		13 (33.33)	
No	2032 (39.00)		133 (27.48)	
Unknown	2,559 (31.71)		291 (29.10)	
**Obesity**		0.002		0.23
Yes	462 (35.03)		28 (33.73)	
No	1781 (39.71)		121 (27.19)	
Unknown	2,477 (31.68)		288 (28.94)	

Medium-term period = three months to one year after the onset of symptoms; Long-term period = one year after the onset of symptoms; COVID-19 immunization = at least 1 dose of COVID-19 vaccine.

Well-separated curves are observed after one year from the onset of symptoms (long-term survival), indicating that survival was worse for individuals who received at least one dose of the COVID-19 vaccine. These results were confirmed in the stratified analysis by number of vaccine doses, shown in the second graph on the right: worse survival occurred in those who took one or two doses compared with those who took no dose (Figure 1).

According to the life table, among the 15,147 survivors after three months of COVID-19, the probability of surviving between the third month post-COVID-19 and the end of the first year was 51 and 15.14% up to two years (Figure 1).

In both periods we observed an excess of deaths among COVID-19 immunized individuals in the Southeastern region and in the urban areas. Specifically in the medium term, there was an excess of deaths among males and females, white people, the Northeast region, in people whose first symptoms occurred in 2021 and 2022, and in hospitalized people. Specifically in the long term, there was an excess of deaths among those with any risk factor, and specifically among those with liver disease (Table 2).

**Table 2:** Death excess (or attenuation) in COVID-19 immunized people by the predictors, Brazil, 2020–2023.

Predictors	Medium-term period				Long-term period			
	Observed	Expected	Excess/ attenuation (%)	*P*-value	Observed	Expected	Excess/ attenuation (%)	*P*-value
Older adult								
Yes	731	710.85	2.84	0.41	107	105.9	−0.86	1.00
No	333	325.72	2.23	0.70	27	27.23	1.03	0.97
Sex								
Female	456	408.39	11.66	0.01	70	55.10	27.05	0.07
Male	608	536.21	13.39	0.001	64	54.42	17.61	0.23
Race								
White	531	463.93	14.46	0.001	69	62.21	10.85	0.45
Black	53	50.78	4.38	0.82	5	3.00	66.67	0.46
Yellow	9	9.20	−2.20	1	0	0.00	0.00	0.13
Mixed race	283	271.75	4.14	0.48	42	34.57	21.48	0.26
Unknown	188	155.36	21.01	0.01	18	13.09	37.54	0.25
Years of study								
Zero	26	32.51	−20.01	0.19	12	6.55	83.33	0.08
1–5	128	112.98	13.29	0.12	21	19.20	9.40	0.80
6–9	72	66.20	8.76	0.49	10	5.83	71.50	0.17
10–12	101	87.71	15.15	0.14	10	10.69	−6.47	1.00
>12	59	48.95	20.54	0.16	4	6.16	−35.01	0.53
Unknown	678	598.80	13.23	0.001	77	63.15	21.93	0.10
Region								
North	43	45.53	−5.57	0.72	9	7.11	26.53	0.63
Northeast	160	137.66	16.23	0.04	30	21.78	37.76	0.1
Southeast	568	477.45	18.97	0.0001	77	58.07	32.59	0.02
South	204	191.79	6.37	0.38	14	20.09	−30.32	0.25
Midwest	89	84.58	5.23	0.66	4	6.21	−35.61	0.5
Area								
Urban	901	790.84	13.93	0.0001	112	90.51	23.74	0.04
Rural	41	41.15	−0.35	1	6	3.41	76.19	0.40
Peri-urban	2	2.63	−23.81	1	0			
Unknown	120	110.36	8.73	0.35	16	14.03	14.01	0.70
Year								
2021	669	568.74	17.63	0.0002	133	132.33	1.00	1.00
2022	340	234.87	44.76	0.0001	0			
2023	55	41.68	32.00	0.42	0			
Hospitalization								
Yes	1,020	908.65	12.25	0.0001	114	101.41	12.41	0.22
No	12	12.24	22.55	0.48	13	4.62	181.67	0.0001
Unknown	29	23.72	22.27	0.32	7	3.71	88.89	0.18
Any risk factor								
Yes	869	834.15	4.18	0.19	102	80.37	26.91	0.02
No	195	152.36	27.99	0.001	32	31.12	2.82	0.97
Heart disease								
Yes	498	479.45	3.87	0.36	51	41.63	22.53	0.16
No	200	184.16	8.60	0.22	21	15.05	39.57	0.23
Unknown	366	308.29	18.72	0.001	62	51.97	19.29	0.21
Diabetes								
Yes	369	338.54	9.00	0.07	40	35.38	13.04	0.49
No	297	275.60	7.79	0.17	29	18.13	59.98	0.03
Unknown	398	347.69	14.47	0.006	65	56.58	8.42	0.32
Kidney disease								
Yes	104	109.21	−4.78	0.58	4	7.62	−47.51	0.18
No	449	409.66	9.60	0.04	48	31.43	52.73	0.01
Unknown	511	442.12	15.58	0.0007	82	70.87	15.69	0.22
Liver disease								
Yes	11	10.77	2.14	1.00	3	1.33	125.00	0.05
No	500	464.87	7.56	0.08	49	35.69	37.32	0.52
Unknown	553	477.39	15.84	0.0003	82	72.65	12.87	0.31
Hemat disease								
Yes	22	15.70	40.16	0.15	3	0.83	260.00	0.39
No	498	466.14	6.83	0.11	49	36.58	33.97	0.07
Unknown	544	471.97	15.26	0.0006	82	71.87	14.10	0.27
Immunodepres								
Yes	63	58.83	7.08	0.62	5	3.53	41.67	0.73
No	469	432.29	8.49	0.06	47	34.35	36.81	0.06
Unknown	532	464.09	14.63	0.001	82	71.84	14.15	0.27
Neurol disease								
Yes	93	93.69	−0.74	1	11	6.81	61.41	0.30
No	448	416.20	7.64	0.09	43	33.34	28.97	0.13
Unknown	523	448.19	16.69	0.0003	80	69.85	14.54	0.26
Down Syndr								
Yes	7	8.00	−12.50	0.88	2	0.00	Inf	0.67
No	510	471.53	8.16	0.06	50	36.34	37.21	0.04
Unknown	547	473.98	15.41	0.0005	82	72.64	12.89	0.31
Asthma								
Yes	32	24.49	30.35	0.14	3	2.50	20.00	1.00
No	495	458.49	7.96	0.07	47	33.96	38.40	0.05
Unknown	537	470.47	14.14	0.001	84	72.76	15.45	0.22
Obesity								
Yes	111	103.12	7.64	0.45	6	7.98	−24.81	0.62
No	427	401.87	6.25	0.18	44	30.73	43.21	0.04
Unknown	526	449.18	17.10	0.0002	84	70.92	18.45	0.15

Medium-term period, three months to one year after the onset of symptoms; Long-term period, one year after the onset of symptoms; COVID-19 immunized, at least 1 dose of COVID-19 vaccine; Immunodepres, immunodepression; Down Syndr, down syndrome; *P*-v = *P*-value.

In the medium-term period, the adjusted analysis indicates a 4 to 8% decrease in the risk of death for those vaccinated. Those who received two doses had 11 to 12% reduction in the risk of death compared to the unvaccinated (reference category), while those who received three doses had 11 to 18% reduction. Adjusted analysis also indicates a 2% increase in the risk of death for each year of life; a 13 to 14% increase in the risk of death for males, a 57 to 70% increase in the risk of death for those with any risk factor; a 22% decrease in the risk of death for those with the higher level of education compared to those without formal education (only in Adjusted Classic Cox analysis), a 8% decrease in the risk of death for non-white (only in Adjusted Classic Cox analysis), and lower risk of death in the Southeast and Northeast, compared to the North (Table 3).

**Table 3:** Crude and adjusted hazard ratio of post-COVID death three months to one year after the symptoms (medium-term effect) according to the predictors (Brazil).

	Crude Cox model	Adjusted classic Cox model ^£^	Adjusted Cox mixed-effects model ^§^	Adjusted Cox fragility model ^¥^
Hazard ratio			Fixed effects	
Main predictors				
COVID-19 immunization	1.12**	0.96 ^NS^	0.92*	0.92*
Vaccine doses				
Zero	1	1	1	1
1	1.24***	1.19^*^	1.13^•^	1.13^•^
2	1.06 ^NS^	0.89*	0.88**	0.88*
3	1.06 ^NS^	0.89^•^	0.82**	0.82*
Covariates				
Age	1.02***	1.02***	1.02***	1.02***
Older adult	1.74***			
Male	1.06*	1.14***	1.13***	1.13***
Race				
White	1	1	1	1
Non-white	0.89***	0.92^*^	0.98 ^NS^	0.99 ^NS^
Unknown	0.87***	0.94 ^NS^	0.96 ^NS^	0.96 ^NS^
Years of study				
Zero	1	1	1	1
1–5	1.00	1.13 ^NS^	1.11 ^NS^	1.11 ^NS^
6–9	0.82*	1.01 ^NS^	1.00 ^NS^	1.00 ^NS^
10–12	0.75**	0.98 ^NS^	0.98 ^NS^	0.97 ^NS^
>12	0.64***	0.78*	0.83^•^	0.83^•^
Unknown	0.65***	0.83*	0.82*	0.82*
Region				
North	1	1		
Northeast	0.83**	0.85**		
Southeast	0.72***	0.70***		
South	1.11^•^	0.98 ^NS^		
Midwest	0.86*	0.87^•^		
First symptoms year				
2020	1			
2021	1.06^•^			
2022	1.03 ^NS^			
2023	1.13 ^NS^			
Hospitalization	1.15 ^NS^	1.05 ^NS^	1.02 ^NS^	1.01 ^NS^
Risk factor	1.97***	1.70***	1.57***	1.57***
Random effects - SD				
City (intercept)			0.47	0.48
ICC			0.06	0.06
Fit measures				
Likelihood ratio		3,386 (df = 18)***	2,852 (df = 402)***	2,861 (df = 59)***
Log-likelihood		- 38706 (df = 18)	−38,111 (df = 343)	−38,087 (df = 364)
AIC		77,447	76,907	76,902
BIC		77,563	79,112	79,243

***p-value < 0.0001; **p-value < 0.001; *p-value < 0.01; ^•^*p*-value < 0.1, NS, not significant; SD, standard deviation; ICC, intraclass correlation coefficient; df, degrees of freedom; AIC, Akaike information criterion; BIC, Bayesian information criterion; COVID-19 immunization, at least 1 dose of COVID vaccine; race unknown, categories unknown and yellow.

To calculate the adjusted effects of COVID-19 immunization, we run two times the same models replacing the variable “COVID-19 immunization” with the variable “vaccine doses”.

^£^ The classic Cox-adjusted model included the following predictors: COVID-19 immunization (or vaccine doses), age, sex, non-white, years of education, region, hospitalization, and risk factors.

^§^ The Cox mixed-effects adjusted model included fixed effects of COVID-19 immunization (or vaccine doses), age, sex, non-white, years of study, hospitalization, and risk factor; and the random effect of the municipality of residence (intercept).

^¥^ The Cox fragility-adjusted model included fixed effects of COVID-19 immunization (or vaccine doses), age, sex, non-white, years of study, hospitalization, and risk factor, and the random effect of the municipality of residence.

In the medium-term period, the standard deviation of the random effects of the Cox mixed effects model was similar to the Cox fragility model (0.47 vs. 0.48) and ICC was the same in these models, 0.06. Likelihood ratio tests in the three adjusted models indicated that the inclusion of covariates was significant. The Adjusted Classical Cox model presented the highest value for the AIC and the lowest for the BIC, which would be expected given that compared to the others, the classical Cox model has more parameters to be estimated. Based on the estimated VIF values for the Adjusted Classical Cox model, all values are close to 1. This suggests that collinearity between the independent variables in your model is low (Table 3).

Figure 2 refers to the classic Cox model adjusted for the medium-term period. It shows no overlap of survival curves for those who took at least one dose of the vaccine and those who did not. We can interpret that the survival experience in the period was worse for those who did not take the vaccine compared to those who took one or more doses. The same figure shows that there is no overlap of survival curves for those who took zero and two doses, as well as between zero and three doses, consistent with the results presented in Table 3. We can interpret that the survival experience in the period was worse for those who did not take the vaccine compared to those who took two or three doses.

**Figure 2:** Post-COVID-19 adjusted Kaplan Meier survival analysis, in the interval between three months and one year after the first symptoms (medium-term effects), according to COVID-19 immunization: at least one dose and number of doses Classic Cox-adjusted model which included the following predictors: age, sex, race, years of education, number of doses of COVID-19 vaccine, region, hospitalization, and risk factors.Brazil, 2020–20,232.

In the long-term period, the adjusted analysis indicates an increase of 4% in the risk of death for each year of life; a decrease of 53% in the risk of death for those with 6–9 years of study compared to those without formal education; risk of death 20 to 25% greater for male; a decrease of 22 to 32% in the risk of death for nonwhite people compared to white ones, a decrease of 45 to 48% in the risk of death for those hospitalized, and lower risk in Midwest region (Table 4).

**Table 4:** Crude and adjusted hazard ratio of post-COVID death one year after the symptoms (long-term effects) according to the predictors (Brazil).

	Crude Cox model	Adjusted classic Cox model ^£^	Adjusted Cox mixed-effects model ^§^	Adjusted Cox fragility model ^¥^
Hazard ratio			Fixed effects	
Main predictors				
COVID-19 immunization	2.06***	1.69***	1.91***	1.94***
Vaccine doses				
Zero	1	1	1	1
1	2.10***	2.02**	2.38***	2.49***
2	2.51***	1.92***	1.97***	1.97***
3	0.97 ^NS^	0.79 ^NS^	0.78 ^NS^	0.76 ^NS^
Covariates				
Age	1.04***	1.04***	1.04***	1.04***
Older adult	3.38***			
Male	0.97 ^NS^	1.20^•^	1.24^•^	1.25*
Race				
White	1	1	1	1
Non-white	0.75**	0.78*	0.70**	0.68**
Unknown	0.70**	0.87 ^NS^	0.66*	0.65*
Years of study				
Zero	1	1	1	1
1–5	0.56*	0.83 ^NS^	0.61^NS^	0.58 ^NS^
6–9	0.41**	0.75 ^NS^	0.49^•^	0.47*
10–12	0.34***	0.73 ^NS^	0.56 ^NS^	0.55 ^NS^
>12	0.33***	0.78 ^NS^	0.50^•^	0.47^•^
Unknown	0.41***	0.85 ^NS^	0.59^•^	0.57^•^
Region				
North	1	1		
Northeast	1.25 ^NS^	1.29 ^NS^		
Southeast	0.94 ^NS^	0.84 ^NS^		
South	1.18 ^NS^	1.03 ^NS^		
Midwest	0.50**	0.56*		
First symptoms year				
2020	1			
2021	2.21***			
2023	27.71***			
Hospitalization	0.54**	0.55**	0.54*	0.52*
Risk factor	1.69***	1.10 ^NS^	1.11 ^NS^	1.14 ^NS^
Random effects - SD				
City (intercept)			0.92	0.91
ICC			0.20	0.20
Fit measures				
Likelihood ratio		541 (df = 18)***	455 (df = 9)***	459 (df = 15)***
Log-likelihood		−2,505 (df = 18)	−2,331 (df = 148)	−2,331 (df = 161)
AIC		5,045	4,959	4,984
BIC		5,118	5,558	5,638

***p-value < 0.0001; **p-value < 0.001; *p-value < 0.01; ^•^*p*-value < 0.1, NS = not significant; SD, standard deviation; ICC, intraclass correlation coefficient; df, degrees of freedom; AIC, Akaike information criterion; BIC, Bayesian information criterion; COVID-19 immunization, at least 1 dose of COVID vaccine; race unknown, categories unknown and yellow.

To calculate the adjusted effects of COVID-19 immunization, we run two times the same models replacing the variable “COVID-19 immunization” with the variable “vaccine doses”.

^£^ The classic Cox-adjusted models included the following predictors: COVID-19 immunization (or vaccine doses), age, sex, race, years of education, region, hospitalization, and risk factors.

^§^ The Cox mixed-effects adjusted models included fixed effects of COVID-19 immunization (or vaccine doses), age, sex, race, years of study, hospitalization, and risk factor; and the random effect of the municipality of residence (intercept).

^¥^ The Cox fragility-adjusted models included fixed effects of COVID-19 immunization (or vaccine doses), age, sex, race, years of study, hospitalization, and risk factor, and the random effect of the municipality of residence.

In the long-term period, the adjusted analysis showed that the risk of death was 69 to 94% higher for those who were vaccinated; and for those who took one and two doses of the vaccine, the risk of death practically doubled compared to those who were not immunized (reference category). For those who took one dose, the risk was 2.02 to 2.49 times higher, and for those who took two doses, the risk was 92 to 97% higher (Table 4).

In the long-term period, the standard deviation of the random effects was similar in the Cox mixed effects model as in the Cox fragility model (0.92 and 0.91, respectively), and the ICC was the same for both modes, 0.20. Likelihood ratio tests in the three adjusted models indicated that the inclusion of covariates was significant. The AIC was higher in the Adjusted Classic Cox model, while the BIC was lower in the Adjusted Classic Cox model, which again would be expected given that compared to the other models, the classical Cox model has more parameters to be estimated (Table 4).

Figure 3 refers to the classic Cox model adjusted for the long-term period. It shows no overlap of survival curves for those who took at least one dose of the vaccine and those who did not. We can interpret that the survival experience during the period was better for those who did not take the vaccine compared to those who took one or more doses. The same figure shows that there is an overlap of survival curves for those who took zero and one dose, as well as between zero and two doses, consistent with the results presented in Table 4. We can interpret that the survival experience during the period was better for those who did not take the vaccine compared to those who took one or two doses.

**Figure 3:** Brazilians post-COVID-19 adjusted Kaplan Meier survival analysis, one year of the first symptoms (long-term effects), according to COVID-19 immunization: at least one dose and number of doses, 2020–2023 Classic Cox-adjusted model which included the following predictors: age, sex, race, years of education, number of doses of COVID-19 vaccine, region, hospitalization, and risk factors.

The analysis of the Martingale residuals for the classic Cox models and the Cox frailty models did not indicate the presence of trends that had not been explained in the adjusted models (data not shown).

## Discussion

In this study, our target population was very specific and vulnerable: all had SARS/COVID-19 and had survived at least three months after the onset of symptoms. Studies have shown a high mortality rate in hospitalized patients, including those in the Intensive Care Unit (ICU), and more than 57% with severe clinical disease of COVID-19 (18–21).

Since the start of vaccination, many studies have reported the benefits of vaccination against COVID-19, including reductions in COVID-19-related hospitalizations, ICU admissions, length of hospital stay, and mortality rates (22–24).

In our analysis, concerning vaccination status, different results were observed between the two periods studied. In the medium-term period, the risk of death decreased among those vaccinated against COVID-19, with a protective effect also for those who received two doses of vaccine and even more for those who received three doses. These results are similar to another Brazilian study that showed the progressive effect of the number of doses in reducing illness severity and death in a cohort of COVID-19 patients, as well as significant improvements in survival after each subsequent dose (2, 4, 22, 25, 26).

Some possible explanations for the reduction in the risk of death in the medium term (after two or three doses of the vaccine) observed in the present study could be: (1) vaccination may be associated with healthier behaviors or greater health awareness (27). For example, vaccinated individuals may be more likely to follow other public health recommendations, such as staying up-to-date with preventive health measures, having regular medical check-ups, or adopting healthier lifestyles. This could lead to a reduction in the risk of death from other causes in the medium term; (2) access to healthcare – since people with comorbidities were prioritized for COVID-19 immunization, these populations may also have benefited from increased medical monitoring and access to healthcare, which may have contributed to a reduction in the risk of death from other causes.

Meanwhile, in the long term, the risk more than doubled for those who received one dose of the vaccine and nearly doubled for those who received two doses. There are two important points to consider: firstly, this is a study that covers all recorded cases of mortality in patients who had SARS/COVID-19 in two periods (medium and long term), and secondly, the analysis of the COVID-19 syndemic in Brazil (28, 29).

Some possible explanations for the increase in the risk of death from other causes in the long term (after one or two doses of the vaccine): (1) adverse effects of the vaccines – while COVID-19 vaccines have proven to be safe for the vast majority of people, there are concerns about potential long term adverse effects (although rare), such as myocarditis, thrombosis, or other rare conditions associated with vaccination (30). These effects may be more pronounced in some groups, particularly in more vulnerable individuals, which could contribute to an increased risk of death from other causes over time; (2) the COVID-19 vaccine may have an indirect effect on the immune system (31, 32) - for people with pre-existing conditions or those with weakened immune systems (such as patients with autoimmune diseases or those on immunosuppressive treatments), the immune response to the virus may have unexpected or complex effects that increase vulnerability to other infections or lead to complications of pre-existing conditions.

According to our findings, in the medium and the long term post-COVID mortality, there was a higher risk in advanced age and men and a lower risk in non-whites. In the medium-term post-COVID mortality, there was a higher risk in those with any risk factor and a lower risk in those with a high level of education. In the long-term post-COVID mortality, there was a higher risk in those with 6–9 years of study, and there was a lower risk in hospitalized people. Several studies have identified social inequality as an important risk factor for mortality in the COVID pandemic showing a significant increase in the mortality coefficient rate of deprived areas (33–40).

All of these studies corroborate to explain that the same aspect that addresses social vulnerability, as seen in our results. In addition, it was observed, in both periods, that there was a higher percentage of deaths in those who had diabetes, heart disease, and kidney disease. We also observed greater percentages in the medium term for neurological disease and Down Syndrome and in the long term for liver disease. This fact emphasizes the concept of the COVID-19 syndemic resulting in the interaction of social iniquities and conditions of vulnerability acting at different levels to increase the effect of COVID-19 (29). Several authors have pointed out the syndemic characteristics of COVID-19 due to its association with the increase of other diseases such as hypertension, diabetes, neglected infectious diseases, obesity, anxiety, and depression, in which there is interaction among them, which potentialize clinical and social impact (29, 37, 39, 40).

The same result was found when we analyzed the mortality risk according to Brazilian regions: the North had a higher mortality risk in both periods, but in the medium term, it was greater than the Southeast and Northeast, and in the long term, it was greater than the Midwest. This can be explained by several social indicators related to education, housing conditions, standard of living, and income distribution, which are better mainly in the Midwest and Southeast compared to the North (41). Other studies have already shown similar results in terms of mortality rate since the beginning of the COVID-19 pandemic in Brazil where these results reflect the geographical and social heterogeneity of the country (1, 42). A study of the effect of socioeconomic inequalities and vulnerabilities on the health system in Brazil (2021) pointed out some relevant points related to (1) The spread of COVID-19 disease in the country: although the state of São Paulo, located in Southeast, had the first confirmed case in the country, the disease rapidly increase of COVID-19 death rates in North and Northeast regions. (2) The analysis of the higher mortality risk in the North was positively correlated with the socioeconomic vulnerability index and inversely, correlated to the health system (37). In an ecological study. Siqueira et al. (43) showed two waves of new cases and deaths during the 18-month COVID-19 pandemic in Brazil. The highest incidence rate was found in the states of Amapá, Rio Grande do Norte, Rondônia, and Roraima, all of which are northern states, except the second, which is a northeastern state. The highest mortality rate was found in the northern states of Amazonas and Rondônia. The authors point out that the regional heterogeneity observed supports the hypothesis that incidence and mortality are related to political, geographical, cultural, and socio-economic factors (43).

The North region has the lowest Gross Domestic Product (GDP) *per capita* in Brazil (44), reflecting the region’s lower urbanization. The North region’s Human Development Index (HDI) is also among the lowest in Brazil (45), reflecting the lower quality of life in terms of education, health, and income. Although there are variations between the states in the region, the HDI of the northern states remains below the national average. It has a vast territorial extension that makes access to health services difficult in rural and isolated areas. In contrast, the Southeast region stands out for presenting high GDP *per capita* and HDI, while the Midwest occupies an intermediate position concerning these indicators. In the Northeast, despite relatively low levels of GDP *per capita* and HDI, urbanization in the Northeast is more advanced than in the North, mainly due to the greater number of large and medium-sized urbanized cities. The Northeast has easier access to health services than the North, especially in urban areas. The Northeast region has a more developed health infrastructure, especially in large cities, and the health system is more accessible in terms of coverage and medical services.

Our target population was patients who had severe clinical disease (SARS) and had comorbidities that were associated with a higher percentage of deaths. The evolution of these comorbidities could therefore not be ruled out as a possible explanation for the increase in post-COVID-19 deaths in the long term. Additionally, it should also be associated with long-term persistence of functional impairment in survivors of severe COVID-19 (SARS), as cited in various studies (46–49). In the long term period, liver disease was also a comorbidity associated with high mortality risk, which could be explained by the liver involvement developed due to COVID-19 disease in hospitalized patients or previous liver disease as reported in a study of systematic review and meta-analysis (50). Moreover, it is important to emphasize that the COVID-19 pandemic provoked a disruption of services and supply chains, access to treatment, and diagnosis as seen before in other periods of economic crisis, in which social determinants were relevant to worse clinical outcomes (51). Furthermore, in the face of the COVID-19 pandemic, the focus has been on the diagnosis and treatment of these cases, to the detriment of other chronic and acute diseases that lead to clinical deterioration and death (52, 53).

Our results indicated a higher risk of post-COVID mortality in whites in the medium and long term. A previous study that we published indicated that the highest risk of short-term mortality occurred mainly in blacks and mixed races (1). Some of the possible explanations could be: (1) after the most intense crisis of the pandemic, a greater number of non-whites had already died (short-term mortality), leaving a surviving population with a lower mortality rate in the following years; (2) although comorbidities are prevalent in both racial groups, the immediate impact of COVID-19 on non-white populations may have resulted in earlier mortality among those who already had preexisting conditions and were more vulnerable. On the other hand, whites who survived the initial infection due to factors, such as better access to health services among others, may have had a greater long-term impact due to other factors, such as comorbidities associated with more advanced aging (given that the white population, on average, has a higher life expectancy). In this study, the protective effect against mortality in non-whites was found in all long-term analyses and only one of the medium-term analyses.

We find no significant increase in the excess deaths among COVID-19-immunized individuals among the older adult. However, we found an excess of deaths among immunized in the Southeast both in the medium and long term and in the Northeast only in the medium term. A publication with 2020 data points to an excess of deaths from ill-defined causes, with the Northeast being one of the regions with the highest excess of deaths (54). A publication with data from 2020 and 2021 detected an excess of deaths in all Southeast states, also highlighting the increase of ill-defined causes of death (55).

In the long term, comparing vaccinated and unvaccinated people, our study found that the risk of death can double in vaccinated people. Serious adverse effects of vaccination cannot be excluded as an explanation of these results, although they are considered to be rare (5, 25, 26, 56, 57). About 0.0042% of serious adverse events were reported by the CDC Vaccine Adverse Event Reporting System (VAERS) (5). The adverse effects/events are associated with each branch of vaccines. A review published that the main serious adverse events were: Cerebral thrombose, Guillain-Barré syndrome (GBS), acute transverse myelitis, Myocarditis and Pericarditis, and Glomerular disease. Cerebral thrombose has been associated with Ad26.COV2.S (Janssen) and AZD1222 (AstraZeneca), both of which use the adenovirus-vector platform and within 28 days of vaccination. GBS - one case was reported a case 11 days after her initial dose of the AZD1222 vaccine, and another case two weeks later after her initial dose of the BNT162 vaccine. Transverse myelitis - three cases in the trial phase of the recombinant AZD1222 vaccine. According to the CDC, more than 10,000 reports of myocarditis were reported to the VAERS after COVID-19 vaccination (Pfizer-BioNTech and Moderna) in the US. The majority of the confirmed cases have been in teenagers and young adults 16 years or older and were often seen after receiving the second dose of the vaccine. The majority of vaccine-related cases were typically seen within one to three weeks after vaccination, especially after the administration of the mRNA vaccines (58). Unfortunately, in the present study, data regarding the type of vaccine and the variation in time between doses are not available in SIVEP, which makes it impossible to analyze any adverse effects related to immunization.

Studies pointed out an association between vaccination against COVID and a small increase in cardiac mortality, especially among men (59), and others, found no evidence of a positive or negative association between vaccination against COVID-19 and an increase or reduction in mortality from all causes (60). It is important to note that this does not necessarily mean that there is a causal relationship with the vaccination. It remains to be elucidated whether it is coincidental or causal (2).

On the other hand, a longitudinal study, post-authorization, showed that even the serious COVID-19 vaccine side effects were rare (0.3%) and highlighted the factors associated with side effects: full vaccination dose, vaccine brand, younger age, female sex, and having had COVID-19 before vaccination (26). In our study, over the long term, those who received one or two doses of the COVID-19 vaccine had a higher risk of death.

According to OMS and based on scientific evidence, the Brazilian Minister of Health adopted the terminology “post-covid conditions” to describe a range of new, recurrent, or persistent clinical manifestations present after acute SARS-CoV-2 infection, when these are not attributed to other causes. These included neurological, cardiovascular, psychopathological, musculoskeletal, gastrointestinal, sleep and sensory disorders. Therefore, there was a possibility that these factors were a confounding element related to factors associated with vaccination (14).

Nevertheless, there is a huge gap in our knowledge of the adverse effects of mass vaccination in a real-life setting, as expected in the long term, and further studies will be undertaken to elucidate the underlying biological mechanisms and identify causality.

## Strengths and limitations

This study stands out for its use of robust survival analysis to assess the risk of post-COVID death. Survival analysis provided a detailed and dynamic view of the impact of the predictors on mortality over time. In addition, the application of different adjusted models (classical Cox, mixed-effects Cox, and frailty Cox) allowed an in-depth analysis of the associations between COVID-19 vaccination and the risk of post-COVID death over different periods. These models are particularly powerful because they not only control for important variables (such as age, sex, race, education, comorbidities, and hospitalization) but also address the complexity of real-world epidemiological data, including variation across locations. These methodological points make the study more reliable and capable of providing insight into the association of different factors with the risk of post-COVID death, helping to inform public health policies and prevention strategies in the medium and long term.

All data were collected from the Sistema de Vigilância Epidemiológica (SIVEP) information system from 2020 to 2023. These cases were likely extremely severe and these patients were also particularly frail given that more than one-third of them died in the post-COVID period. This raises the possibility of a strong selection bias in trying to evaluate possible factors associated with it. As an example, if vaccination had a strong impact (as suggested in tons of well-done studies) on reducing the risk of severe diseases and COVID-19 deaths, this study selection is looking only at those patients for whom vaccination did not provide a benefit and then is measuring the risk in a wrong way.

This study focused on just the most serious cases of COVID-19, classified as Severe Acute Respiratory Syndrome, and therefore does not reflect the total magnitude of cases and deaths from COVID-19 in Brazil. These cases were likely extremely severe and these patients were also particularly frail, which reduces the inferential scope of our results.

The completeness of data for some notification fields that are not mandatory generates a significant loss of information. In addition to unfilled data, fields marked as “ignored” also reduce the possibility of evaluating variables.

Unfortunately, the Brazilian system for reporting adverse events from vaccines, including against COVID-19 [Post-Vaccination Adverse Events Information System (SI-EAPV)], is not open access, which makes it difficult to obtain accurate information on this issue in Brazil.

Due to the need to only include cases of death after acute COVID-19, we made sure to include in this study all deaths that occurred three months after the first symptoms of COVID-19. Issues of incorrectly filling out the cause of death on the death certificate could make it impossible to detect the real panorama of post-COVID deaths in Brazil, for this reason, we chose to include all deaths that occurred, regardless of the cause.

Due to the lack of access to some information, this study did not consider some aspects such as the types of vaccines, the intervals between the onset of COVID-19 symptoms and vaccination, and between vaccination and death.

Unfortunately, few Brazilian studies evaluated post-covid mortality, which makes it difficult to assess the consistency of the results found in this study, however, the strength of association shown in our results indicates the need to expand this field of investigation.

## Conclusion

This study delves into the complex dynamics of post-COVID mortality risk, particularly concerning vaccination, in the Brazilian context from 2020 to 2023. Notably, it acknowledges the multifaceted nature of COVID-19, with various factors influencing mortality risk, including age, gender, race, schooling, comorbidities, and vaccination status.

The study goes further to investigate the long-term impact of vaccination on mortality, revealing a nuanced picture. Although immunization against COVID-19 confers protection against mortality in the medium term, our results indicate the possibility that the effect reverses in the long term.

Notably, the study highlights demographic disparities in mortality risk, with advancing age, male gender, and the presence of comorbidities being associated with higher mortality. These findings are consistent with previous research and underscore the importance of targeted interventions for vulnerable populations.

Overall, this study contributes valuable insights into the complex interplay between vaccination, demographic factors, and mortality risk in the context of COVID-19. However, it also underscores the need for further research to fully understand the long-term implications of vaccination and to inform ongoing public health strategies.

## Data Availability

The original contributions presented in the study are included in the article/supplementary material, further inquiries can be directed to the corresponding author.
